# Changes in Humans' Autonomic Nervous System under Dynamic Lighting Environment During A Short Rest

**DOI:** 10.1155/2021/6697701

**Published:** 2021-08-20

**Authors:** Chien-Yu Chen, Pei-Jung Wu, Yu-Jen Hsiao, Yu-Wen Tai

**Affiliations:** ^1^Graduate Institute of Color and Illumination Technology, National Taiwan University of Science & Technology, Taipei 10607, Taiwan; ^2^Center for General Education, National Taichung University of Science and Technology, Taichung 40401, Taiwan; ^3^Department of Neurology, National Taiwan University Hospital Yunlin Branch, Yunlin 64002, Taiwan; ^4^Department of Electronics Engineering, National Yunlin University of Science and Technology, Yunlin 64002, Taiwan

## Abstract

Overloaded work and life stress often result in excessive fatigue and stresses in people, further leading to psychological burden and physiological disease. In this case, good rest is important in busy life. Good rest could result in good quality of life and work efficiency. In order to assist people in getting into deep rest to obtain a restorative state after fatigue, a dynamic lighting system with low-frequency change for assisting users in effective relaxation is proposed in this study. Heart rate variability analysis is used for discussing the change in the autonomic nervous system of the subjects under dynamic lighting environment, and a self-report questionnaire is applied to understand the subjects' psychological feeling. The research results indicate that the subjects significantly showed enhancement in the activities of parasympathetic nervous system within 25 minutes in the dynamic lighting process, in comparison with the steady lighting system. The questionnaire survey results also reveal that the subjects receive higher quality of rest, after the dynamic and low-illuminance lighting stimuli, with good feeling.

## 1. Introduction

In the modern society with information overload, overtime work and high-stress life often result in people's negative feelings of fatigue, stress, and loss. Excessive fatigue and stress could easily result in psychological burden leading to psychological diseases of anxiety and depression [1, 2]; physiological diseases, such as destroyed physiological rhythm, endocrine disorder, and insomnia would also occur [3, 4]. For this reason, it is urgently required for modern people to understand how to effectively release fatigue and stress. Rest is an option for many people beating fatigue. This research found out the important effect of good rest on life and work [5]. Nevertheless, what would be good rest? Long-time rest is not certainly good rest; good rest refers to people being with enough comfort. A theoretical definition of rest includes a beneficial state that is intentional, temporary, and restorative when people have problems such as physical and mental work or activity, fatigue, trauma, illness, or stress [6–8].

Light could show visual impact and nonvisual effects on humans, and it could tightly influence the autonomic nervous system. Light pulse could enter suprachiasmatic nuclei (SCN), through the retina and retinohypothalamic pathway, as the biochemical signal transduction [9, 10], to induce the autonomic pathways in the hypothalamus to regulate humans' response of autonomic nervous system. Humans' internal clock could induce activity or regeneration through external light; e.g., improving the subjects' attention and sleep impulse with bright light which, as phototherapy, could even improve the elderly depression [11–13]. Moreover, external light could induce humans' internal rhythm through oscillation [14] to affect the change in humans' autonomic nervous system. Autonomic nervous system (ANS) is a component of the peripheral nervous system, which could control human functions of heartbeat, blood pressure, and respiration with reflex action. ANS is divided into sympathetic nervous system and parasympathetic nervous system. Sympathetic and parasympathetic nervous systems of healthy people would resist each other to achieve the balance [15]. Research indicated that the activities of parasympathetic nervous system in the autonomic nervous system would increase when people feel relaxed and comfortable [16]. Nevertheless, when people felt fatigue and bore excessive stress, the secretion of corticosteroids would increase to enhance the activities of sympathetic nervous system, and the activities of parasympathetic nervous system would relatively reduce and make people hardly get into relaxation that rest could not achieve the relaxing effect [17].

According to the above literature, this study proposed a system with dynamic and low-illuminance lighting with low-frequency change to assist users in effective relaxation, expecting to actually help people get into deep rest to obtain a restorative state after the fatigue. The effects of steady lighting environment and dynamic lighting environment on humans' autonomic nervous system and psychological feeling within a certain period are discussed in this study. Accordingly, heart rate variability [18] is regarded as the objective indicator for evaluating the subjects in the experiment. The changes in the activities of sympathetic nervous system and parasympathetic nervous system of the subjects with distinct luminous environment stimuli could be understood through the frequency parameter change in heart rate variability. Furthermore, a self-report questionnaire is also used as the subjective indicator for evaluating the subjects' psychological feeling.

The research results indicate that the activities of parasympathetic nervous system of the subjects in the dynamic lighting process proposed in this study, compared to the steady lighting system, significantly increase in 25 minutes. The questionnaire results also reveal that the subjects receive higher rest quality, after receiving the dynamic and low-illuminance lighting stimuli, with good feeling. The above results show that the dynamic and low-illuminance lighting system proposed in this study indeed could assist people in efficient rest and relaxation. The research would be applied to people with different needs in the future, e.g. people in graveyard shift, people frequently back and forth different time zones, and even patients in long-term care centers and long-hour workers.

## 2. Materials and Methods

### 2.1. Design of Experiments

This study aims to discuss the change in the subjects' autonomic nervous system in short rest, under the dynamic and low-illuminance lighting environment, in 3 groups that are arranged for the experiment. Group Control is the control group, in which the subjects rest without light stimuli; the subjects in Group SLI rest under the steady and low-illuminance (10 lux) lighting environment; and the subjects in Group DLI rest under the dynamic and low-illuminance lighting environment. To avoid the effect of circadian rhythm on the experimental result [19, 20], the experiment is preceded during 7 PM to 9 PM. The experiment process is shown in Figure 1. The experiment time for each group is 1.5 hours, merely a group of subjects execute the experiment for a day, and the sequence for participating in the experiment is random.

In the beginning of the experiment, the subjects have to proceed with 20 mins of dark adaptation, 50 mins of luminous environment stimuli, and 20 mins of the questionnaire survey. During the 50-minute short rest time with different environments, subjects sit on a recliner and relax their mood and bodies. The electrocardiogram signals of the subjects are measured in the first 70 minutes. This study is in accordance with the Declaration of Helsinki and is examined and verified by Research Ethics Committee National Taiwan University, with the approval case number 201807EM029.

### 2.2. Experimental Environment

The three experimental groups in this study are arranged in different luminous environments. After the first 20 mins of dark adaptation, the subjects in Group Control stay in the environment without lighting. Steady and low-illuminance (10 lux) white light with the color temperature about 2750 K, as the home rest environment, is used as the luminous environment for Group SLI, and dynamic and low-illuminance (10 lux-0.05 lux) lighting environment is designed for Group DLI. According to the literature [21], the red spectrum could better go through eyelids than other visible spectra. The dynamic lighting environment therefore is designed mainly with the red spectrum (LED main band 630 nm); nevertheless, monochromatic light is comparatively uneventful such that little different spectra are used for mixing light to modulate the soft dynamic color spectra. The dynamic light period is 90 seconds, as shown in Figure 2. In order to not affect melatonin secretion, the illuminance in the luminous environment in this study does not exceed 10 lux [22].

An adjustable multichannel LED lighting system (LED Cube, THOUSLITE) is used in the experiment to simulate the abovementioned steady and dynamic lighting. The light is at a distance of 1 m from the subjects, and the illuminance received by the subjects' eyes is about 10 lux. The experiment environment is shown in Figure 3, and the temperature in the experiment environment is controlled at 26 ± 1°C.

### 2.3. Subjects

A total of 21 healthy subjects (6 females and 15 males), with the average age of 23.9 ± 0.9, participate in the experiment. These subjects do not suffer from sleep disorder and cardiovascular disease and do not have a history of drug use. Besides, tea, coffee, alcohol, and smoking, which might affect heart rhythm, are not taken 8 hours before the experiment [23–26].

### 2.4. Analysis of Heart Rate Variability

Heart rate variability (HRV) is used as the indicator to evaluate response of the autonomic nervous system in this study. HRV is the method to test heart rate changes. The international standards announced by the European Society of Cardiology and North American Society of Pacing and Electrophysiology in 1996 clarify the correlations between research on the autonomic nervous system with HRV and various physical and mental diseases [18]. According to the standards, the changes in HRV parameters and the corresponding response of the autonomic nervous system of the subjects resting under distinct luminous environment are tested in this study.

In the experiment, Biopac MP150 (model ECG 100C, AcqKnowledge; Biopac Systems, Santa Barbara, CA, USA), a multifunctional physiological measuring instrument, is used for recording Lead II electrocardiogram signals of the subjects. Each electrocardiograph characteristic peak *R* is extracted from the subjects' electrocardiograph records, and the interval between peaks is regarded as the R-R interval. Abnormal R-R intervals resulted from arrhythmia and atrial fibrillation are removed in this study. 5 mins is taken as a unit of the ECG segment for monitoring the changes of HRV on the subjects during the short rest. The detailed information is shown in Figure 4. According to the standard measurement of HRV [18], a short-term HRV analysis should use at least a value of 512 for 5-minute recordings. In this study, subjects start to have a short rest for 50 mins after the dark adaptation in each group. Each 5-minute segment at 5^th^ minute, 10^th^ minute, 15^th^ minute,…, 45^th^ minute during the short rest is measured for HRV analysis. Every segment contains at least 512 R-R intervals and the R-R interval time series must be an even-sampled time series. In addition, it is needed to detect and remove the artefacts because FFT analysis is highly sensitive [27, 28]. After the above process, the R-R interval data are interpolated and resampled at a 4 Hz [29, 30] for FFT.

In the HRV spectrum, the frequency of total power (TP) ranges from 0.01 Hz to 0.4 Hz, the frequency of high-frequency power (HFP) ranges from 0.15 Hz to 0.4 Hz, the frequency of low-frequency power (LFP) ranges from 0.04 Hz to 0.15 Hz, and the frequency of very low-frequency power (VLFP) ranges from 0.01 Hz to 0.04 Hz. HFP is the indicator of the activities of parasympathetic nervous system in the human autonomic nervous system, and LFP is the comprehensive indicator of the activities of sympathetic nervous system and parasympathetic nervous system. LFP and HFP in this study are normalized for nLFP and nHFP:

(1) $$\begin{array}{c} nLFP=\frac{LFP}{TP-VLFP}, \end{array}$$

(2) $$\begin{array}{c} nHFP=\frac{LFP}{TP-VLFP}. \end{array}$$

Related research indicated that people would show excitement and anxiety when the activities of sympathetic nervous system increased but would be more relaxed when the activities of parasympathetic nervous system increased [31]. Accordingly, the changes of activities of sympathetic nervous system and parasympathetic nervous system of the subjects in the same groups and under the same luminous environment are analyzed.

### 2.5. Subjective Evaluation

Subjective evaluation is also applied in this study to evaluate the subjects' actual feelings under distinct luminous environment. A 6-point self-report questionnaire and short qualitative interview are used for the evaluation; the questionnaire items are shown in Table 1. The comfort of the experiment space, the relaxation of the subjects, and the spirit conditions of the subjects are discussed in the questionnaire. The higher point reveals the higher agreement. After the questionnaire survey, a short qualitative interview is preceded, mainly for understanding the subjects' other feelings about the work and living habits not listed in the questionnaire items.

### 2.6. Statistical Analysis

In terms of statistical analysis, SigmaStat statistical software (SigmaStat statistical software, Jandel Scientific, San Rafael, CA, USA) is used for analyzing the HRV parameters and questionnaire results of the groups. To understand the subjects' response of autonomic nervous system change with time, under distinct luminous environment stimuli, repeatedly measure ANOVA with Student–Newman–Keuls tests of HRV parameters is utilized for in-group statistical analyses. Between-group statistical analyses of HRV parameters are not proceeded for comparing the results of 3 groups, because the experimental environments in this study contains not only one single light factor. Many Group Control ANOVA with Student–Newman–Keuls tests is applied to compare the questionnaire results among 3 groups in order to realize the subjects' actual feelings after the experiment.

## 3. Results

Figure 5 shows the nLFP and nHFP changes on the subjects in three experimental groups.  Figure 5(a) shows that nLFP of the subjects in Group Control does not show obvious changes with time and the mean appears to be 26.7 ± 1.7. nHFP slightly increases in 20 mins, but not obvious, and the mean is revealed to be 39.4 ± 2.4.  Figure 5(b) displays that nLFP of the subjects in Group SLI under the steady lighting environment does not show obvious changes with time and the mean appears to be 39.7 ± 2.0.  Figure 5(c) shows that nLFP of the subjects in Group DLI under the dynamic lighting environment does not reveal obvious changes with time and the mean value is 26.3 ± 2.4. Nonetheless, the nHFP mean of 49.7 at the 25^th^ minute is significantly higher than the mean of 34.5 at the 5^th^ minute, with statistical difference (*p* < 0.05). The nHFP mean of 48.5 at the 30^th^ minute is apparently higher than the mean of 34.5 at the 5^th^ minute, with statistical difference (*p* < 0.05).

The questionnaire analysis results are shown in Figure 6, where the subjects consider most relaxation in Group DLI under the dynamic lighting environment, with the evaluation point 4.3 ± 0.9. In comparison with Group SLI under the steady lighting environment and Group Control, the subjects in Group DLI could better relax, with statistical difference (*p* < 0.05). On the other hand, there is no statistical difference in the evaluation of better spirit after the experiment. Nevertheless, the subjects in Group DLI feel better spirit, with the evaluation point 4.6 ± 0.8. Finally, the 3 groups do not show statistical difference in the comfort of environment and the evaluation points do not show obvious differences.

## 4. Discussion

According to the HRV analysis result, the subjects in Group DLI with dynamic lighting reveal significantly increasing nHFP in the first 30 minutes and the significant differences appear on the 25^th^ minute and the 30^th^ minute; however, the nLFP do not show significant changes during light stimuli. It reveals that the activities of parasympathetic nervous system of the subjects present obvious increase in the 30 mins of stimuli of low-illuminance environment with low-frequency change. The activities of parasympathetic nervous system of the subjects in Group Control appear slight increase, but not remarkable difference. The activities of sympathetic nervous system and parasympathetic nervous system of Group SLI with steady lighting do not reveal notable difference. Literature studies indicated that people's activities of the parasympathetic nervous system in the autonomic nervous system would increase when feeling more relaxed [31]. In comparison with the other two groups, the dynamic lighting environment proposed in this study indeed could efficiently enhance users' activities of the parasympathetic nervous system and allow users achieve the relaxation within 30 minutes. On the other hand, the questionnaire results discover that the subjects feel more relaxed under dynamic lighting environment, significantly higher than in Group Control and Group SLI. After the dynamic lighting experiment, the subjects' spirits are better than the other two groups, but without statistical difference. In regard to the comfort of environment, the subjects in three groups do not feel significant difference in the experiment environment. The study reveals that the subjects would not feel uncomfortable or inadaptable in low-illuminance environment with low-frequency change. In summary, the activities of parasympathetic nervous system of the subjects under dynamic and low-illuminance lighting remarkably increase and the subjects feel better relaxed that the results of the objective evaluation are consistent with the results of the subjective evaluation.

Different light stimuli, such as color, brightness, duration of exposing in luminous environment, oscillation, and illumination time, might result in distinct physiological reactions of different ethnic groups. Single light factor would present various effects on the autonomic nervous system of different ethnic groups. Moreover, effects of the complex factor in light stimuli might not show consistent effects on the autonomic nervous system. For instance, exposure under blue luminous environment presents calm and relaxation functions [32, 33]; however, excessive short-wavelength blue light in the evening would affect humans' circadian rhythm and response of the autonomic nervous system causing insomnia [22, 34]. Since there are not complete and systematic findings on the effect of different light stimuli on humans' physiological mechanism and the luminous environment for the 3 groups in this study is not one single light factor, the changes in the activities of sympathetic nervous system and parasympathetic nervous system of the subjects under distinct luminous environment are not discussed when comparing the results of the response of autonomic nervous system of the three groups. Different light stimuli would be separated into various but constant single light factors in the future to analyze and discuss the effect of dynamic lighting on the autonomic nervous system.

According to the literature [14], humans' internal rhythm could be induced by external light with oscillation to influence the change in humans' autonomic nervous system. The frequency change of the dynamic and low-illuminance lighting system proposed in this study is within humans' ultradian rhythms [35]. Vincent Grote et al. considered that light oscillation with ultradian rhythms could help achieve the optimal autonomic balance and body regulation [36]. Human health, with great extent, relied on the state and balance of the autonomic nervous system [15, 18]. When people felt excessive fatigue or stress, the activities of sympathetic nervous system revealing excitement for a long period could easily disorder the autonomic nervous system [17]. The research results show that dynamic and low-illuminance lighting could effectively enhance users' activities of the parasympathetic nervous system in a short time with better relaxation psychologically. It is therefore inferred that dynamic lighting could improve light or temporary autonomic nervous system disorder. The application would be expanded to the field with long working hours or unfixed working hours, e.g., people in graveyard shift, people frequently back and forth different time zones, and even patients in long-term care centers and long-hour workers, in the future research. Furthermore, it would be an interesting and meaningful issue whether such dynamic lighting systems could be applied to clinics as phototherapy for improving patients' autonomic nervous system disorder.

## 5. Conclusions

A dynamic lighting system with low-frequency change to assist users in effective relaxation is proposed in this study, HRV analysis is used for discussing the change in the subjects' autonomic nervous system in the use process, and a self-report questionnaire is applied to understand the subjects' psychological feeling. The research results indicate that the activities of parasympathetic nervous system of the subjects under the dynamic and low-illuminance lighting, compared to the steady lighting system, show significant increase, and the subjects feel more relaxed. The result of the objective evaluation is therefore consistent with the result of the subjective evaluation. The study would be applied to people with different needs, such as people in graveyard shift and frequently back and forth different time zones and even patients in long-term care centers and long-hour workers, in the future.

## Figures and Tables

**Figure 1:** Experimental processing.

**Figure 2:** The designed dynamic lighting in this study.

**Figure 3:** Experimental environment.

**Figure 4:** The detected R-R interval information during the short rest.

**Figure 5:** The variation of normalized low-frequency power and high-frequency power in (a) Group Control, (b) Group SLI, and (c) Group DLI during the short rest (^*∗*^*p* < 0.05).

**Figure 6:** The subjective results from the questionnaire (^*∗*^*p* < 0.05).

**Table 1:** The content of the questionnaire.

	Item	1	2	3	4	5	6
1	You feel comfortable about the experiment space.						
2	You are relaxed in the short rest.						
3	You are in better spirit after short rest.						

## Data Availability

The data used to support the findings of this study are available from the corresponding author upon request.
